# Bioinformatics facilitating the use of microarrays to delineate potential miRNA biomarkers in aristolochic acid nephropathy

**DOI:** 10.18632/oncotarget.10586

**Published:** 2016-07-13

**Authors:** Yana Lv, Yumei Que, Qiao Su, Qiang Li, Xi Chen, Haitao Lu

**Affiliations:** ^1^ Key Laboratory of Dai and Southern Medicine of Xishuangbanna Dai Autonomous Prefecture, Yunnan Branch, Institute of Medicinal Plant Development, Chinese Academy of Medical Sciences, Peking Union Medical College, Jinghong 666100, P.R. China; ^2^ Shanghai Center for Systems Biomedicine, Key Laboratory of Systems Biomedicine (Ministry of Education), Shanghai Jiao Tong University, Shanghai 200240, P.R. China; ^3^ Innovative Drug Research Centre and School of Chemistry and Chemical Engineering, Chongqing University, Chongqing 401331, P.R. China; ^4^ Tissue Repair and Regeneration Program, Institute of Health and Biomedical Innovation, School of Biomedical Sciences, Faculty of Health, Queensland University of Technology, Brisbane 4059, Australia

**Keywords:** aristolochic acid nephropathy, microRNAs, network biology, functional analysis, biomarkers

## Abstract

Aristolochic acid nephropathy (AAN) is a rapidly progressive acute or chronic tubulointerstitial nephritis (TIN). The present study attempted to explore the molecular mechanisms underlying the miRNA-directed development of AAN. Our differentially expressed analysis identified 11 DE-miRNAs and retrieved the target genes of these DE-miRNAs; then, network analysis and functional analysis further identified 6 DE-miRNAs (has-miR-192, has-miR-194, has-miR-542-3p, has-miR-450a, has-miR-584, has-miR-33a) as phenotypic biomarkers of AAN. Surprisingly, of has-miR-192 has been reported to be associated with the pathogenesis of AAN, and has-miR-194, has-miR-542-3p and has-miR-450a was first-time identified to link to the development of AAN. In addition, the expressional changes of has-miR-584 and has-miR-33a may be associated with the development of AAN as well, which must be further confirmed by the associated experiments. Taken together, our work reveals for the first time the regulatory mechanisms of miRNAs in the development of AAN and this will contribute to miRNA-based diagnosis and treatment of AAN.

## INTRODUCTION

Aristolochic acid nephropathy (AAN) is a rapidly progressive acute or chronic tubulointerstitial nephritis (TIN) that occurs during end-stage renal failure and urothelial malignancy [1]. Patients taking aristolochic acid have a high risk (~50%) of upper urothelial tract carcinoma as well as bladder urothelial carcinoma within a few years; such cases have occurred in Europe and Asia [2, 3]. The predominant lesion of AAN is characterised by tubulointerstitial fibrosis, with tubular atrophy atrophy/loss and global glomerular sclerosis [2, 4, 5]. Apoptosis, epithelial-mesenchymal transition (EMT), and fibrosis are the main pathologic manifestations of the development of AAN. DNA damage, cell cycle arrest, and cell apoptosis have been studied in an AA-induced proximal tubular epithelial cell line (LLC-PK1) as well as proximal tubular epithelial cells (PTCs). Inflammation is also one of the mechanisms involved in AAN. TGF-/Smad3 may play a critical role in AAN. A previous study by Zhou et al [6]., found that AA could activate Smad signalling to mediate EMT and renal fibrosis through TGF-dependent and JNK/MAP kinase-dependent mechanisms. p53 is involved in the apoptotic injury seen in AAN. Previous studies also showed that AA stimulated the p53 pathway, mediating TEC apoptosis in acute AAN [7, 8]. Moreover, AA-DNA adducts are an AA exposure marker and risk factors of AA nephropathy-associated cancer [9]. AA commonly induces tumours in the renal cortex, renal pelvis and urinary bladder. Furthermore, some tumours have also been discovered in the forestomach, lungs, uterus and lymphoid organs [10]. However, the underlying pathogenesis of AAN remains largely unclear, which has impeded the development of effective therapies for AAN patients. Currently, a synthesize assay method is urgently needed that can identify the targets of AAN, and What 's more, explore molecular mechanisms of AAN, is necessary.

In disease network, system biology concentrates on complex molecular interaction, instead of changing single molecular component. Network biology analysis can discovery individual molecular component has little affect disease network. Network pharmacology, which is based on system biology and polypharmacology, provides a novel dominant paradigm for drug design that encompasses the network mode of “multiple targets, multiple effects, complex diseases” [11, 12]. Interestingly, research ideas of network pharmacology is correspond with the holistic and systemic views of Traditional Chinese medicine (TCM) [13, 14]. TCM network pharmacology provides a comprehensive analysis for TCM Formula, and TCM-based drug discovery [15]. For example, Li shao et al [16]., employed a network pharmacology method to identify bioactive ingredients and action mechanisms of Ge-Gen-Qin-Lian decoction for Type 2 Diabetes therapy. Moreover, network pharmacology can speculate and appraise toxicity and side effects of drugs by adopting the network analysis strategy. Thus, network pharmacology has become a powerful tool for identifying drug target, and then uncovering the therapeutic and toxicological mechanisms of TCM formulae. This shall promote modern study and development of TCM.

MicroRNAs (miRNAs) are a class of small (~22 nucleotides) non-coding RNAs that regulate gene expression by causing translational repression or degradation of target mRNA at the post-transcriptional level [17, 18]. miRNAs play key roles in a variety of biological process, such as cell apoptosis, proliferation, differentiation, development and tumorigenesis, and are involved in the development of many diseases, including cancer, nephropathy and renovascular diseasesuch as cell apoptosis, proliferation, differentiation, development and tumorigenesis, and involved in development of many diseases including cancer, nephropathy and renovascular disease [19–21]. Many studies have found that miRNAs play a role in the progression of renal disease. For example, miR-34a suppresses renal cancer cell growth, tube formation and metastasis [22], and miR-24 promotes renal ischemic injury by inducing apoptosis in endothelial and tubular epithelial cells [23]. However, few previous studies have emphasised the value of circulating miRNAs as potential biomarkers for AAN therapy.

In the study, network pharmacology method was employed to unwind miRNA complexity in the progression of AAN. First, we analyzed the miRNA expression profiles from HK-2 normal samples and HK-2 samples treated with AA to identify DE-miRNAs using microarray analysis, and further the target genes of DE-miRNAs were predicted. Next, we performed a network analysis and functional analysis of these DE-miRNAs to uncover their roles in the progression of AAN. Finally, 6 DE-miRNAs (has-miR-192, has-miR-194, has-miR-542-3p, has-miR-450a, has-miR-584, has-miR-33a) were screened as potential biomarkers for AAN therapy. Our results may provide novel insight into the regulatory mechanisms of miRNAs in the progression of AAN and be useful for the prevention and treatment of AAN.

## RESULTS

### Screening of DE-miRNA

After preprocessing, we obtained miRNA expression data that composed of 6 samples and1222 miRNAs. The miRNA expression data was analyzed using SAM. According to the threshold of FDR<0.05, we identified 11 DE-miRNAs. The information for 11 DE-miRNAs were listed in Table 1.

**Table 1:** Eleven differentially expressed miRNAs

No.	miRNA	Fold change
1	hsa-miR-33a	6.59
2	hsa-miR-450a	5.99
3	hsa-miR-194	6.30
4	hsa-miR-192	8.35
5	hsa-miR-4730	5.26
6	hsa-miR-542-3p	5.19
7	hsa-miR-4747-3p	4.21
8	hsa-miR-1234	4.51
9	hsa-miR-584	6.27
10	hsa-miR-3663-3p	5.11
11	hsa-miR-3135b	4.20

Note: FDR<0.05.

### Construction of differentially expressed miRNA-gene regulation networks and miRNA-pathway regulation networks

To increase the reliability of the predicted DE-miRNA targets, we selected target genes that were stored in at least five databases. We predicted the target genes of each DE-miRNA and constructed a network using Cytoscape (Figure 1). The miRNA -gene regulation network consisted of 988 nodes for target genes, 7 nodes for DE-miRNAs, and 1074 regulatory relationships between 7 DE-miRNAs and 988 target genes. The yellow squares represent miRNA. Based on the numbers of DE-miRNAs regulating the target genes, the target genes are represented as bright green, light blue, orange and red circles. In the network, we observed certain target genes that were regulated by more than one miRNA. For example, GPR158 were regulated by hsa-miR-450a, hsa-miR-194, hsa-miR-584, and hsa-miR-33a.

**Figure 1:** Regulatory network of differentially expressed miRNA-genes In the miRNA-gene regulation network, yellow squares denote miRNAs. Target genes are represented in bright green, light blue, orange and red circles based on the number of regulatory relationships between the miRNAs and target genes. Bright green indicates one regulatory relationship, light blue denotes two regulatory relationships, orange denotes three regulatory relationships, and red indicates four regulatory relationships.

We performed pathway enrichment analysis of DE-miRNA target genes using the hypergeometric distribution test. Biological pathways with significant values (p<0.05) were identified as significant pathways. We identified the significant pathways for each DE-miRNA and built a miRNA-pathway regulation network using Cytoscape (Figure 2). In the network, 92 nodes were significant pathways, 6 nodes were DE-miRNAs, and 138 edges represented the regulatory relationships between significant pathways and DE-miRNAs. The DE-miRNAs are shown as yellow squares and the coloured circles denote target genes in light blue, pink, green and red based on the number of regulatory relationships between the miRNAs and target genes. Figure 2 shows that the pathways associated with inflammatory and immune functions were regulated by miRNAs, such as cytokine-cytokine receptor interactions, Wnt signalling pathways, MAPK signalling pathways, NOD-like receptor signalling pathways, B cell receptor signalling pathways and T cell receptor signalling pathways. Additionally, 12 cancer-related pathways were also represented, specifically prostate cancer, basal cell carcinoma, pathways in cancer, glioma, renal cell carcinoma, endometrial cancer, acute-myeloid leukaemia, colorectal cancer, pancreatic cancer, melanoma, small cell lung cancer, and non-small cell lung cancer. Furthermore, cell cycle, calcium signalling pathway, p53 signalling pathway, insulin signalling pathway, apoptosis, and others were also significantly regulated by miRNAs.

**Figure 2:** Regulatory-network analysis of miRNA-pathways In the miRNA-pathway regulation network, yellow squares represent miRNAs, and the coloured circles denote pathways in light blue, pink, green and red based on the number of regulatory relationships between significant pathways and miRNAs. Light blue represents one regulatory relationship, pink represents two regulatory relationships, green represents three regulatory relationships, and red represents four regulatory relationships.

Given the miRNA-gene regulation network and the miRNA-pathway regulation network (Figures 1 and 2), information about the degrees of DE-miRNAs is shown in Figure 3; we found that has-miR-194 (305 genes and 15 pathways) had the greatest number of links to adjacent target genes, and has-miR-33a (230 genes and 43 pathways) had the greatest number of connections to adjacent pathways. Other miRNAs, including hsa-miR-542-3p (243 genes and 42 pathways), hsa-miR-584 (175 genes and 24 pathways), hsa-miR-192 (104 genes and 14 pathways), and hsa-miR-450a (17 genes and 1 pathways), also had connections with adjacent target genes and pathways.

**Figure 3:** Information for the degrees of the DE-miRNAs In the two networks, the degrees represent the numbers of connections between miRNAs and target genes/pathways.

### Functional analysis of target genes of DE-miRNA

We performed GO biological process (BP) annotation analysis of DE-miRNA target genes using the hypergeometric distribution test. The GO terms with significant values (p<0.05) were identified as GO biological process. We identified the significant GO terms for each DE-miRNA and plotted the distribution of the GO biological process annotations (Figure 4). GO terms for hsa-miR-192, hsa-miR-542-3P, and hsa-miR-450a that were classified as biological processes by WEGO. The biological process terms suggested that hsa-miR-192 and hsa-miR-542-3p were mainly correlated with biological regulation, cell cycle, cellular metabolic process, cellular process, metabolic process, and others (Figure 4A. The biological process terms suggested that hsa-miR-33a, hsa-miR-194, and hsa-miR-584 are mainly involved in biological regulation, cellular metabolic process, cellular process, metabolic process, pigmentation (Figure 4B).

**Figure 4:** Distribution of the GO terms for the target genes of DE-miRNAs **A.** The GO terms for the target genes of hsa-miR-192, hsa-miR-542-3P, and hsa-miR-450a were classified into biological process by WEGO. **B.** The GO terms for the target genes of hsa-miR-33a, hsa-miR-194, and hsa-miR-584 were classified into biological processes by WEGO.

## DISCUSSION

In the study, we employed bioinformatics methods to identify 6 DE-miRNA(has-miR-192, has-miR-194, has-miR-542-3p, has-miR-450a, has-miR-584, and has-miR-33a) in AAN, which could better our understandings of the pathogenesis of AAN and provide potential biomarkers for diagnosis and treatment. miRNAs perform a complex role in cell cycle arrest induced by the increased activation of p53, which is a major feature of AAN [24, 38–40]. The miR-192 and miR-194 affect cell cycle progression, which is induced by p53 [41–44]. Jenkins et al [24]., noted the over-expression of has-miR-192, has-miR-194, has-miR-450a and has-miR-542-3p in AA-induced G2/M arrest in proximal tubular epithelial cells (PTCs), and our study indicated that the has-miR-192over-expression is recapitulated in G2/M arrest in AAN. has-miR-194 was significantly up-regulated in acute kidney impairment and down-regulated in the growth arrest injury in carcinogenesis; for example, miR-194 is often down-regulated in colorectal cancer, renal childhood neoplasms, and multiple myeloma [45–48]. Previous studies have indicated that the expression of has-miR-194 may cause G1 and G2 arrest in a p53-dependent manner [41, 43]. The above studies suggested that altered has-miR-194 expression is most likely to contribute to the progression of AAN. miR-542-3p is a tumour suppressor that improves p53 stability by promoting the regulatory relationship between p53 and MDM2, a negative regulator of p53 [49]. Yoon et al [50]., demonstrated that the enforced expression of miR-542-3p caused the inhibition of cell proliferation and apoptosis by inducing G1 and G2/M cell cycle arrest. has-miR-450a targeted the MAPK signalling pathway in HK-2 cells treated with AA, and the MAPK signalling pathway results in the fibrosis that accompanies the tubular atrophy/loss that is the main lesion in AAN [51–53]. Moreover, has-miR-450a was reported to be significantly decreased in hepatocellular carcinoma as well as ectopically; its expression leads to cell proliferation inhibition through DNMT3a [54]. has-miR-33a is a tumour suppressor that inhibits cell cycle progression [55]. A previous study found that miR-33a transfection led to reduced cell proliferation in colon carcinoma cells, and miR-33a inhibition increased cisplatin-induced apoptosis by antagomir-33a in osteosarcoma cells [56, 57]. Additionally, miR-33a inhibits expression of the insulin receptor substrate 2, which is involved in the insulin-signalling pathway in the liver [58]. miR-584 has been reported to be inhibitd in kidney cancer and breast cancer [59, 60].miR-584 has anti-inflammatory effects that modulate AA functions [61]. Subsequently, miR-584 regulated pathways such as MAPK signalling pathways, pathways in cancer, Wnt signalling pathways, p53 signalling pathways, and TGF-beta signalling pathways are associated with AAN [9, 53, 62–66]. Thus, has-miR-33a and has-miR-584 may be biomarkers for the diagnosis and prognosis of AAN, which must be confirmed in further experiments.

In addition, MDM2 is target gene for has-miR-192, has-miR-194, and has-miR-542-3p. It was shown that the expression of MDM2, a negative regulator of p53, was suppressed by AA, while has-miR-192 was significantly up-regulated. The analysis suggested that over-expression of has-miR-192 resulted in G2/M cell cycle arrest by inhibiting MDM2 expression via the increased activity of p53. In AAN, the expression of MDM2 is down-regulated, but has-miR-192 is over-expressed in renal cells after AA treatment, indicating that MDM2 is related to cell cycle and AAN-associated cancers [4]. RB1 is target gene for has-miR-192. RB1 is a tumour suppressor gene and a negative regulator of the cell cycle [67, 68]. A study by Chang [69]., suggested that AA-induced urothelial proliferation in rats via cell-cycle progression was mediated via the induction of cyclin D1/cdk4 and/or cyclinE/cdk2 activity and the increasing phosphorylation of Rb. Volker et al [70]., also confirmed that RB1 is often affected in human urothelial cancer. CDC7 is the G1 and G2 checkpoint protein of has-miR-192 and contains has-miR-194. It encodes a cell division cycle protein with kinase activity that is critical for maintaining genomic stability via the S-phase checkpoint pathways in response to DNA damage, which can be associated with AAN [4].

This study has some limitations. First, the retrieval of miRNA target genes may not have been complete. Although we retrieved target genes of miRNAs based on 10 databases, the identified target genes might include false positives. Second, current material on AAN-related miRNAs is limited, and their regulatory mechanisms in the development of AAN are still largely unclear. Third, the sample sizes for the expression profiling were not large. We hope that additional high-throughput data can be obtained. Despite these limitations, the study still provides insight into miRNA regulation in the developmental process of AAN.

## MATERIALS AND METHODS

### Microarray analysis

The miRNA expression profile of GSE53911 was downloaded from the GEO database (http://www.ncbi.nlm.nih.gov/geo/), which was amassed by Jenkins et al [24]. A total of six human proximal tubular epithelial cell line (HK-2) samples were selected, including 3 HK-2 cells without AA treatment (used as controls) and 3 HK-2 cells with AA treatment. The annotation information of for the miRNA expression profiles was downloaded from the GPL15446 3D-Gene Human miRNA V17_1.0.0 platform.

### Data preprocessing

For the miRNA expression profiles, we first inferred missing values using the K-nearest neighbours method [25]. Then, these values were normalised with the limma package in R [26]. The probe level data were finally converted into miRNA names based on the annotation information from the GPL15446 platform.

### Differentially expressed miRNAs analysis

To identify the differentially expressed miRNAs (DE-miRNAs), a significance analysis of microarrays (SAM) was used to screen the DE-miRNAs, and miRNAs with a false discovery rate (FDR) threshold of less than 0.05 were designated as differentially expressed.

### DE-miRNA target genes prediction

The target genes of DE-miRNA were retrieved from the following miRNA-target databases:DIANA-microT(DT) [27], mirSVR [28], PicTar5(PT5) [29], RNA22 [30], RNAhybrid(Rh) [31], TargetScan (TS) [32], PITA [33], MirTarget2 [34], TargetMiner [35], miRanda (miR) [36]. Target genes were identified in at least 5 out of the 10 databases to decrease the number of false-positive results.

### Pathway and functional analysis

We performed pathway and functional analyses for the target genes of each DE-miRNA using the hypergeometric distribution test which can identify significant pathways and GO biological processes. The p value for each pathway or GO term was calculated as follows:

$$\text{p}=1-\sum_{\text{i}=0}^{\text{m}}\frac{\begin{array}{cc} \text{M} & \text{N}-\text{M}\\ \text{i} & \text{n}-\text{i} \end{array}}{\begin{array}{c} \text{N}\\ \text{n} \end{array}}$$

where N denotes the total number of the whole human genome, n is the number of DE-miRNA target genes, M represents the number of genes that are annotated to a pathway or a GO term, and m is the number of annotated DE-miRNA target genes in a pathway or a GO term. Pathways or GO terms with p<0.05 were considered to be significantly enriched and could be regulated by DE-miRNA. We plotted the distribution of the GO annotation using WEGO (http://wego.genomics.org.cn/cgi-bin/wego/index.pl) [37].

## CONCLUSIONS

In our study, we first performed differentially expressed miRNA analysis and identified 11 DE-miRNAs associated with AAN. Next, we performed network analysis and functional analysis on the target genes of these DE-miRNAs. Finally, 6 DE-miRNAs (has-miR-192, has-miR-194, has-miR-542-3p, has-miR-450a, has-miR-584, and has-miR-33a) were predicted as potential biomarkers of AAN. has-miR-192 has been shown to be involved in the pathogenesis of AAN. The altered expression of has-miR-194, has-miR-542-3p and has-miR-450a appear to link to the progression of AAN, but how they exert the regulatory effects in AAN progression is still not clear. has-miR-584 and has-miR-33a have known roles in the progression of cancer and can affect the development of AAN. Although these targets were selected, there have not been many reports that have clearly explored their roles, and further studies are need to confirm their roles in AAN progression. Moreover, the genes MDM2 and RB1 were identified as being significantly affected in AAN-urothelial cancer, and the gene CDC7 was identified as being associated with AAN. However, further investigation is required to confirm the function of CDC7.
